The article "Adolescent Psychological Assistance Treatment Strategy Integrating Home-School Coordination and Network Information" was retracted in 2024. Reasons: signs of a paper mill; suspected computer-generated content; unreliable results or conclusions; lack of ethics approval or compliance.

# Adolescent Psychological Assistance Treatment Strategy Integrating Home-School Coordination and Network Information

**DOI:** 10.1155/2022/6393139

**Published:** 2022-07-14

**Authors:** Yaling Li

**Affiliations:** Mental Health Education and Counseling Center, Shenzhen Technology University, Shenzhen, 518118 Guangdong, China

## Abstract

With the continuous satisfaction of material life, teenagers' physical health has been generally improved, and all aspects of competition have posed a challenge to teenagers' mental health. Therefore, both at the family level and at the school level, teenagers' mental health education has been paid more and more attention. The school cooperative education model came into being, which has had an important impact on the mental health education of teenagers. Family education is the first level of education for teenagers. Parents' role model, family education concept, and education model all play a key role in the development of children's mental health. Based on this, this paper will focus on optimizing the home-school cooperation strategy, further clarify the main responsibilities of the school, teachers, and parents in the home-school cooperation education in the strategy, establish and improve the home-school cooperation mechanism based on this, and focus on the cultivation of parents' mental health education and teachers' mental health guidance professional skills in this process. Based on the current situation of network home-school mental health coordination and mental health education, this study takes teenagers as the research object, aiming at the common psychological problems in learning, social adaptation, and interpersonal communication, and tries to study the problems of promoting teenagers' mental health from the perspective of integrity and development. The developed home-school collaboration method is to verify that the network home-school collaboration method is more effective than the traditional home-school collaboration method in promoting the mental health development of primary school students, so as to provide a reference for the theory and practice of home-school collaboration under the network environment to carry out mental health education. According to the corresponding network information intelligent algorithm, this paper constantly adjusts the coordination strategy between family and school and guides teenagers to internalize the corresponding excellent behaviour into their own habits. In the experimental part, the psychological assistance treatment scheme proposed in this paper is verified and analysed. The experimental results show that the psychological assistance treatment program for adolescents proposed in this paper has obvious effects. School education has a special mental health counseling center and special psychological teachers, which can carry out mental health education more scientifically. The unity and cooperation between family education and school education can combine the educational power of parents and schools to fully develop the mental health of teenagers.

## 1. Introduction

Adolescent mental health diseases have become an important factor affecting the healthy development of adolescents. Serious mental health problems affect adolescents' daily life and learning, and even intervene in their judgment of the world, thus forming abnormal and distorted values and world outlook [1–3]. Most of the common mental health problems of teenagers are caused by the external environment, which often lacks the corresponding psychological guidance and education; therefore, timely intervention and treatment for the mental health problems of teenagers and timely intervention and treatment through drugs or psychotherapy will play a good role in improving the mental health status of teenagers. At present, the traditional mental health assistance treatment for adolescents is mainly carried out by improving improper cognition, correcting their behavior and habit errors and drug treatment, but lack of active intervention of the external environment and intervention and improvement of information technology [4–6]. In the speech therapy programs such as improving improper cognition and correcting their behavior habit errors, the mainstream traditional programs include psychosocial therapy mode and conversation mode therapy. The main treatment processes are as follows: first, mainly understand the mental and psychological conditions of patients from the social level and then, from the psychological dynamics, conduct a comprehensive analysis on the causes of mental health problems and the corresponding patients at the physiological level, and finally, provide a comprehensive, multilevel, and multiangle treatment scheme for adolescent patients [7, 8]; at the corresponding drug treatment level, the current main drug treatment includes mild drug treatment and severe drug treatment, and the main drug used is psychotropic drugs. In addition to the above treatment schemes, the corresponding cognitive behaviour treatment scheme is also popular and reliable, but this treatment scheme is usually combined with drug treatment for comprehensive treatment. Its specific treatment schemes include exposure treatment scheme, self-cognitive change scheme, muscle training relaxation scheme, and social learning treatment scheme. Based on the above analysis, the traditional treatment scheme for adolescent psychological problems is often too single and does not have the function of self-renewal and self-adaptation. Therefore, it does not have the characteristics of keeping pace with the times and personalization. Therefore, the proposal of the new treatment scheme has epoch-making significance [9, 10].

As one of the important interactive measures of adolescent psychological assistance treatment program, home-school system strategy mainly emphasizes the collaborative role of family therapy and school therapy and emphasizes the mutual dependence and promotion between them, to optimize the problems existing in current adolescents to the greatest extent [11, 12]. At the level of teenagers' psychological problem assistance, home-school collaboration solves the linkage problem between home and school to a certain extent and makes a breakthrough analysis on Teenagers' psychological problems from two levels, to ensure the solution of teenagers' psychological problems in different environments [13–15]. However, the traditional home-school collaboration mechanism has problems such as single structure and unclear collaboration subject. The subject object of home-school collaboration is only limited to the literal school and home and has not been further extended to society, community, and even groups, which reduces the advantages of home-school collaboration mechanism to a certain extent [16–18]. At the same time, the communication in the traditional home-school coordination mechanism also has serious efficiency problems. Generally, the communication mechanism between school and family is extremely narrow, the corresponding communication channels are single and poor, and the information between family and school is also lack of timeliness and reliability. Therefore, there is a serious disconnection between the corresponding family education and school education [19, 20].

Based on the above research on the current situation of adolescent psychological assistance treatment and home-school coordination mechanism, the following conclusions are drawn: adolescent mental disease has become an important factor affecting the healthy growth of adolescents, which has brought great trouble to adolescents' life and learning, and is easy to cause the lack of personality at the same time. The traditional adolescent mental health assistance treatment is only limited to conversation and drug treatment and rarely uses modern information means for adjuvant treatment. At the same time, the traditional home-school coordination strategy has the phenomenon of single structure and lack of subject in adjuvant psychotherapy. Based on this, this paper proposes to optimize the traditional home-school collaboration strategy, clarify the main responsibilities of teachers and parents in home-school collaboration education, establish and improve the home-school collaboration mechanism, and pay attention to parent education and the cultivation of teachers' professional skills. Under the background of the optimized home-school coordination mechanism, this paper will also improve the communication mode of home-school coordination based on the corresponding network information technology, through the guidance of network information, and continuously adjust the coordination strategy between home and school according to the corresponding network information intelligent algorithm, to provide a reasonable way to relieve pressure and vent for teenagers, so as to improve teenagers' self-cognitive ability and guide teenagers to internalize the corresponding excellent behaviour into their own habits. In the experimental part, the psychological assistance treatment scheme proposed in this paper is verified and analysed. The experimental results show that the psychological assistance treatment scheme for adolescents proposed in this paper has obvious effect and popularization significance.

Based on the above comprehensive analysis, the structure of this paper is arranged as follows: the second section of the article will mainly analyse the research status of adolescent psychological assistance treatment based on network information under the home-school coordination strategy and analyse its main problems and causes; the third section of this paper will mainly analyse and study how to carry out psychological assistance treatment for teenagers based on network information under the optimized home-school coordination strategy and formulate treatment plans based on relevant theories; the fourth section of this paper will select the corresponding samples for the experiment based on the treatment scheme of this paper, analyse the experimental results, and improve the treatment scheme proposed in this paper; finally, this paper will summarize and give the follow-up research plan.

## 2. Related Research: Analysis of the Research Status of Adolescent Psychological Assistance Treatment Based on Network Information under the Home-School Collaborative Strategy

A large number of scholars and research institutions have conducted research and analysis on adolescent psychological assistance. First of all, at the level of adolescent psychological assistance treatment, the current mainstream research includes drug therapy, cognitive behavior therapy, play therapy, and team psychological counseling [21–23], and the corresponding treatment methods are also diverse, mainly in a single way or in a combination of multiple ways. In terms of corresponding drug treatment level, relevant Japanese scholars believe that juvenile mild psychosis can be treated. The experimental results show that this treatment method has good curative effect [24]. This method is mainly used for drug intervention treatment of juvenile patients with mild mental diseases, which is essentially a physical treatment method; for cognitive behaviour therapy, scholars in Chinese Mainland believe that self-confidence training can help patients change their social psychology and help them provide help at the psychological level. This method advocates psychopsychological intervention rather than physical therapy. European and American scholars have proposed to realize the psychological assistance treatment for adolescent patients based on sand table games, mainly providing personalized services based on sand table games, so as to improve the frequency of teenagers' communication with the outside world, improve the quality of communication with people, and alleviate certain anxiety. This experimental scheme has a good effect on improving teenagers' psychological problems. This method mainly intervenes teenagers' psychological diseases through behavioral therapy, and this method has certain contingency. However, with the continuous improvement of social informatization, the related social problems are becoming more and more prominent, and the traditional psychological assistance treatment scheme for adolescents has little effect. Therefore, relevant scholars combine it with the home-school cooperation strategy. However, the traditional home-school cooperation strategy and adolescent psychological assistance research are too limited to theoretical analysis and lack of corresponding practice and suggestions. Therefore, such treatment schemes are not feasible [25–28]. Based on the above analysis, there are many urgent problems to be solved in the current adolescent psychological assistance treatment.

## 3. Analysis and Formulation of Psychological Assistance Treatment Plan for Teenagers Based on Network Information under the Home-School Coordination Strategy

This section mainly discusses the formulation and analysis of adolescent psychological assistance treatment scheme based on network information under the strategy of school collaboration. The corresponding treatment scheme is shown in Figure 1. It can be seen from the figure that the specific scheme includes the analysis and investigation of specific teenagers' psychological problems and growth, the diagnosis and analysis of problematic teenagers' psychological problems, the analysis of the causes of psychological problems, the classified diagnosis and analysis of their physiological, psychological and social adaptability, the formulation of treatment assistance scheme based on the collaborative background of home and school, and the optimization of their treatment scheme by means of network information implementing the corresponding treatment plan. In the whole treatment plan, the corresponding psychological status diagnosis includes dynamic diagnosis and static diagnosis. The corresponding dynamic diagnosis includes the diagnosis and analysis of teenagers' id, ego, and superego. At the same time, the dynamic diagnosis also includes the influence of family environment and related factors; at the level of corresponding cause diagnosis, we need to analyse the causes of the problems, and deeply analyse the growth environment and adverse factors of individuals when they were young; the corresponding classification and diagnosis level mainly includes the personality at the psychological level, the sleep at the physiological level and the treatment at the social adaptation level; at the level of formulating treatment assistance programs corresponding to the background of home-school collaboration, the main analysts analyse the background of home-school collaboration, fully optimize the current problems of home-school collaboration strategies, and formulate corresponding treatment programs based on this; at the level of optimizing the treatment plan by means of network information, the self-adaptive optimization of adolescent psychological assistance treatment plan is mainly realized based on network information technology; in the final implementation stage of the program, the concerted efforts of families, schools, and society are needed to jointly promote the implementation of the program, integrate the ideas and abilities of the school, parents and teachers in the home-school collaboration strategy, analyse the responsibilities and abilities of the school, teachers, and parents in the guidance and analysis of adolescent mental diseases, further clarify their corresponding optimization direction based on their needs' abilities and responsibilities, and provide demand support for the systematic proposal of home-school collaboration strategy.

### 3.1. Analysis of Psychological Assistance Treatment Scheme for Adolescents Based on Network Information under Home-School Coordination Strategy

This section mainly analyses the discussion of the details of the scheme adopted in this paper. The main discussion contents include the optimized home-school cooperation strategy and the implementation of network information assistance technology.

For the psychological problem assistance of teenagers, the home-school coordination strategy needs to be further optimized to solve its disadvantages. The corresponding problems and the corresponding optimization strategy are shown in Figure 2. As can be seen from Figure 2, the corresponding optimization strategies are as follows: society, schools, and families should pay attention to teenagers' mental health problems, schools should establish exclusive files for teenagers with mental health problems, and the corresponding file contents should cover the teenagers' school information and family information, to facilitate schools and families to have a full understanding of them, clarify the main responsibility status of the school under the home-school coordination strategy, determine the corresponding problem youth objects that need to be served, clarify the treatment objectives, clarify the corresponding school treatment plan, and realize the clear division of labor between the school and the family at the same time; establish a long-term and effective home-school coordination mechanism to ensure the long-term development of adolescent mental health assistance; schools should pay attention to the cultivation of teachers' ability in the home-school cooperation mechanism. Its main abilities include the cultivation of cooperative concept, cooperative communication ability, cooperative experience summary and reflection ability, and the cultivation of teachers' personal quality; help to improve the ability of parents, cultivate parents to become the main body of home-school coordination strategy, help parents establish correct values and cultivation outlook, guide parents to provide assistance and treatment for teenagers' internal psychological problems, and help parents actively cultivate a good family relationship with teenagers.

### 3.2. Under the Strategy of Home-School Coordination, Psychological Assistance, and Treatment Plan for Adolescents Based on Network Information

Based on the above optimization of home-school coordination strategy, this section formulates the psychological assistance treatment scheme based on the optimization strategy. The corresponding specific scheme is shown in Figure 3. It can be seen from the figure that the corresponding scheme mainly includes the determination of responsibility, the confirmation of long-term and scientific home-school coordination mechanism, the support mechanism of information network technology, the cultivation of teachers' responsibility and ability, and the cultivation of family education responsibility and ability, reflection, summary, and optimization.

As can be seen from the figure, the specific implementation details of the scheme proposed in this paper are as follows:

At the level of determining the responsibility subject, it mainly includes determining the responsibilities of schools, teachers, and parents, determining the treatment objects and objectives of the adolescent psychological assistance treatment plan, and clarifying the content of psychological health assistance treatment, to further formulate the psychological assistance treatment strategy, implement the psychological health assistance treatment plan, and finally, realize the implementation of the psychological assistance treatment plan. In this process, the school should first help parents understand the seriousness of teenagers' mental health problems and the necessity of psychological assistance treatment and actively guide parents to transform teenagers' bad mental state into normal mental state. At this stage, the school should also make a specific analysis of teenagers' personality, family factors, and family status according to their specific conditions, to put forward targeted opinions and treatment strategies. In the specific implementation process, it is necessary to further clarify the relevant responsibilities of schools, families, and teachers and carry out fine division of labor.

At the level of determining the corresponding long-term and scientific home-school coordination mechanism, we should first clarify the long-term effectiveness, sustainability, and scientificity of the corresponding mechanism. In the third stage, we need to rely on network information technology to establish an effective storage mechanism. Based on this storage mechanism, we can improve the timeliness and efficiency of home-school cooperation scheme, and rely on network information technology to store a large amount of timely data. At this stage, the corresponding home-school coordination mechanism and the corresponding scheme need to be sound and comprehensive. The corresponding sound mainly refers to the sound and comprehensive content of home-school coordination education, the comprehensive and reliable home-school coordination feedback mechanism and the reliable and effective evaluation level of home-school coordination mechanism.

In terms of the supporting mechanism of the corresponding information network technology, this paper mainly realizes the real-time communication and analysis of the corresponding home-school cooperation based on the wireless sensor network. Through the cloud storage mechanism, the real-time data and recorded data of teenagers' mental health status under a large number of home-school collaborative strategies are stored and transmitted. Based on the real-time monitoring and communication of adolescent mental health, the home-school collaborative linkage analysis and monitoring are mainly based on real-time network communication tools.

At the corresponding teacher level, the cultivation of responsibility and ability mainly includes the cultivation of teachers' concept of home-school collaborative analysis of adolescent mental health, teachers' communication ability, teachers' experience summary, and reflection ability. At the corresponding level of teachers' cultivation of the concept of home-school collaborative analysis of adolescent mental health, it mainly emphasizes the importance and necessity of adolescent mental health assistance and emphasizes the guiding role of teachers. At this level, it is necessary to cultivate teachers' awareness of home-school collaborative service and cultivate their corresponding dedication and selfless dedication; at the corresponding level of the cultivation of teachers' communication skills, it is necessary to cultivate the participation of teachers' collaborative strategies at this level, so that the mental health problems of teenagers in school can be reflected in time and received corresponding attention. By cultivating teachers' communication skills, schools and parents can form a certain joint force, to better implement home-school collaborative strategies and better solve the problem of adolescent mental health assistance; at the corresponding level of cultivating teachers' experience summary and reflection ability, schools can regularly carry out home-school collaborative education seminars on adolescent mental health assistance and cultivate teachers' experience summary and reflection ability in the form of seminars. Based on this seminar, teachers are encouraged to share their experience in home-school collaborative strategies for adolescent mental health assistance and reflect on the problems existing in the strategies in time, promote learning exchanges between teachers, and promote an atmosphere of mutual learning.

At the corresponding level of family education responsibility and ability training, first of all, we need to help parents establish the awareness of home-school coordination of adolescent mental health assistance, clarify that parents, as an important link for schools to solve adolescent mental health problems, need to actively assist schools in adolescent mental health assistance and estimate that parents pay more attention to adolescent mental problems, cognitive problems, and the establishment of values; actively assist parents to increase their knowledge of home-school collaboration and information network technology, improve their comprehensive literacy in psychology and mental health assistance, put forward guiding opinions on adolescent mental health assistance under home-school collaboration strategy based on this, enrich their corresponding knowledge, and finally, realize the thinking interaction between parents and schools; assist parents to establish a good parent-child relationship, guide teenagers to express their feelings through parents, get out of the haze, actively solve mental health problems, help parents establish a positive and optimistic sense of responsibility in details, and help them realize the importance and necessity of communication, to make corresponding teenagers with mental health problems feel happy and happy; assist parents to establish a good image of positive, influence teenagers imperceptibly through parents, and set an example for teenagers.

In the corresponding reflection summary and optimization part, it is mainly based on the in-depth learning algorithm in information network technology to continuously learn and optimize the specified scheme through feedback data and evaluation. Aiming at the mental health problems of different teenagers, considering their personality, family situation, and physiological situation, we formulate the mental health assistance treatment scheme under the cooperation of home and school and make iterative optimization and improvement according to the treatment level of different stages. The corresponding technical framework of reflection and summary based on network information technology is shown in Figure 4.

Based on the above home-school coordination strategy, the formulation of psychological assistance treatment plan for teenagers based on network information can give full play to the advantages of home-school coordination strategy and make full use of information network technology to continuously optimize and improve the treatment plan, so as to realize the sustainability and effectiveness of the treatment plan.

## 4. Experiment and Data Analysis

Based on the above formulation of adolescent mental health assistance treatment plan, this section carries out the experiment based on the experimental sample data and analyses and summarizes the experimental data. The main experimental object is a group of problem teenagers with a sample of 20 people. Through this experiment, we provide assistance treatment for their mental health problems. The main experimental design is shown in Figure 5.

The main experimental evaluation indicators of the experimental part include the improvement of teenagers' mental health problems (quantitative analysis through psychological test scores), the cultivation of teachers' home-school collaborative ability (the main evaluation indicators include concept awareness, communication ability and teachers' experience summary and reflection ability), and parents' awareness ability (the main evaluation indicators include parents' awareness).

Through the psychological assistance treatment of the sample 20 people, the main responsibility of the treatment subject is the school, teachers, and parents. At the same time, through long-term treatment, the treatment effect was improved. Finally, the treatment effect was evaluated by the corresponding psychological test scores. The score comparison table of the corresponding 20 people before and after treatment is shown in Table 1, and the corresponding comparison line chart is shown in Figure 6. It can be seen from the chart that through the treatment scheme proposed in this paper, the corresponding psychological problems of problem adolescents have been improved to a certain extent, and the psychological problems have been improved. At the same time, it can be seen from the table that the adolescents with low scores mean that their corresponding mental health problems are serious. Through the treatment of this scheme, their corresponding scores are increased by about 30%, which shows that their mental problems have been greatly improved.

At the same time, this paper carried out experimental verification at the level of home-school collaborative optimization, which mainly verified the improvement of teachers' and parents' ability. The experimental results of this part are mainly investigated and analyzed in the form of questionnaires, and the corresponding optimization conclusions are obtained through the statistical analysis of the questionnaires. As shown in Figure 7, the comparison chart of teachers' abilities before and after the implementation of the scheme is shown. The main comparative indicators include the main evaluation indicators (including concept awareness, communication ability, teachers' experience summary, and reflection ability). As can be seen from Figure 7, through the implementation of the home-school collaboration strategy proposed in this paper, the collaboration ability of parents and schools has been improved by about 20% compared with the traditional strategy. The ability of teachers and parents to guide and sort out the corresponding psychological problems has been further improved, and the home-school collaboration strategy has been guaranteed.

The corresponding Figure 8 is a column diagram of parents' improvement in consciousness and ability before and after treatment. It can be seen from the figure that the home-school collaborative optimization strategy proposed in this paper plays an important role in improving the ability of parents. Compared with the home-school collaborative strategy before optimization, parents have made great progress in home-school collaborative awareness, home-school collaborative knowledge reserve and efficient communication with their children.

Based on the above experimental results, the adolescent psychological assistance treatment scheme based on information network under the home-school coordination strategy proposed in this paper has obvious advantages, and it has obvious significance for the treatment of adolescent psychological problems, the cultivation of school teachers' ability and the cultivation of parents' ability.

## 5. Conclusion

This paper mainly analyzes the research status and existing problems of related concepts such as adolescent mental health assistance and home-school coordination strategies. In order to solve the problems of self-renewal and learning of adolescent mental health assistance programs, this paper optimizes the traditional home-school coordination strategy, clarifies the main responsibilities of teachers and parents in home-school coordinated education, and establishes and improves the home-school coordination mechanism, parent education, and the development of teachers' professional skills. Under the background of the optimized home-school coordination mechanism, this paper improves the communication mode of home-school collaboration based on the corresponding network information technology and the guidance of network information and continuously adjusts the home-school collaboration strategy according to the corresponding network information intelligent algorithm and provides a reasonable way to relieve stress and vent for young people, thereby further improving the self-cognition ability of young people and guiding young people to internalize the corresponding excellent behaviors into their own habits. In the experimental part, the psychological assistance treatment scheme proposed in this paper is verified and analyzed. The experimental results show that the adolescent psychological assistance treatment scheme proposed in this paper has obvious effect and promotion significance. The main research ideas on the home-school collaborative strategy of adolescent psychotherapy in the later stage will focus on a large number of test and verification of sample data, as well as the summary, reflection, and optimization of corresponding schemes. At the same time, this paper will further refine the specific details in the later research, to make the adolescent mental health treatment under the home-school collaborative strategy more standardized. Based on this, the corresponding modifications are highlighted in the conclusion part of the article.

## Figures and Tables

**Figure 1:** Framework of psychological assistance treatment scheme for adolescents based on network information under the home-school coordination strategy.

**Figure 2:** Guiding framework of current home-school collaboration strategy problem analysis and optimization approach.

**Figure 3:** Framework of psychological assistance treatment scheme for adolescents based on network information under the home-school coordination strategy.

**Figure 4:** Technical framework of reflection and summary based on network information technology.

**Figure 5:** Experimental block diagram of psychological assistance treatment scheme for adolescents based on network information under the home-school coordination strategy.

**Figure 6:** Broken line chart of psychological test scores of sample data before and after treatment.

**Figure 7:** Comparison of teachers' ability before and after the implementation of the scheme in the home-school collaborative ability.

**Figure 8:** Comparison of parents' ability before and after the implementation of the scheme.

**Table 1:** Comparison of sample data and psychological test scores before and after treatment.

Sample serial number	Pretreatment score	Posttreatment score	Sample serial number	Pretreatment score	Posttreatment score
1	77	85	11	55	79
2	65	79	12	68	85
3	78	88	13	79	89
4	67	79	14	78	88
5	66	79	15	77	90
6	70	83	16	67	89
7	78	88	17	54	77
8	45	78	18	34	76
9	47	78	19	66	87
10	77	87	20	32	77

## Data Availability

The data used to support the findings of this study are included within the article.
